This article has been retracted.

# Machine Learning of ZnO Interaction with Immunoglobulins and Blood Proteins in Medicine

**DOI:** 10.1155/2022/4062974

**Published:** 2022-03-16

**Authors:** Nasreddin Abdel Qader Osman, Shatha Hallal Al-Ziyadi, Malik Bader Alazzam, Samar Zuhair Alshawwa, Md Adnan Rahman

**Affiliations:** ^1^College of Mass Communication, Ajman University, Ajman, UAE; ^2^Saudi Board Certified in Obstetrics & Gynecology, Taif University, Taif, Saudi Arabia; ^3^Information Technology College, Ajloun National University, Ajloun, Jordan; ^4^Department of Pharmaceutical Sciences, College of Pharmacy, Princess Nourah bint Abdulrahman University, P.O. Box 84428, Riyadh 11671, Saudi Arabia; ^5^Green Business School, Green University of Bangladesh, Dhaka, Bangladesh

## Abstract

Toxoplasmosis is a zoonotic illness caused by *Toxoplasma gondii*. Those with a normal immune system normally recover without treatment. Immunocompromised individuals and pregnant women must be treated regularly. Toxoplasmosis is a serious illness that may reactivate in immunocompromised patients. A retrospective study using machine learning of toxoplasmosis patients at Government Fever Hospital in Gorantla, Guntur, India, included 25 women, eight of whom were pregnant. These included sex, age, symptoms and side effects, pregnancy, ophthalmic, and antitoxoplasmosis titers, and treatment regimens. Protease mobility and specific activity were increased in toxoplasmosis-infected women's sera, although not significantly (*p=*0.05). However, there was no discernible decline. The impacts of nanoparticle impact demonstrated a 52.24 percent drop in compound concentration in the presence of zinc nanoparticles, whereas the effect of ZnO nanoparticles was 51.37 percent. Zinc nanoparticles lowered IgA, IgG, and IgM levels in the eye.

## 1. Introduction

Nanoparticles are susceptible to interception by several defense components after entering the body due to their size [1], shape, and surface chemistry. Several machine learning that inhibit the shift in perspective processes can be used to make macrophages avoid nanoparticles. Surface modification or coating of nanoparticles with naturally occurring complement inhibitors results in stealth or macrophage-avoiding nanoparticles [2–6]. Toxoplasmosis is caused by *Toxoplasma gundi*, a protozoan with a heterogeneous life cycle that may infect a variety of well-evolved beast and poultry species through diverse transmission paths, with cats serving as the authoritative host [7]. It has a global reach; serological tests have revealed a wide variety of effects, affecting a wide range of countries, geographic areas, and ethnic groups. Although the tachyzoite form of the parasite must be demonstrated histologically or by [8–12] the isolation procedures to make a definitive diagnosis of toxoplasma infection and toxoplasmosis, advances in serologic diagnosis have largely eliminated the need for biopsy and isolation studies, except in a few patients with congenital toxoplasmosis and when disease occurs in patients who are immunocompromised the machine learning of nanotechnology in the therapy, prevention, and management of underlying biological illnesses is referred to as nanomedicine [13–16]. To employ nanomedicine, the precise cellulitis target (cells and receptors) must be discovered, and the appropriate nanoparticles for delivery methods must be chosen to limit the effects of the first treatment. Nanoparticles (NPs) are a type of particle that may be utilized to target specific tissues or cell types with drugs or diagnostics. Their potential application in toxoplasmosis research and treatment as well as in breaking down the immune system is particularly intriguing. They are a strategy for increasing pharmacological data such as drug release, organ specificity, and even cell specificity, in theory. Nanomaterials include quantum dots, liposomes, nanospheres, carbon nanorods, and nanotubes as well as zinc, gold, palladium, and magnet NPs. The most commonly used elements in the recent ten years were zinc, silver, and gold NPs, which accounted for the majority of articles. Using a similar concept of NP conjugation with parasite biomarkers, more parasitic illnesses were discovered. In the case of toxoplasmosis, the application of selective agglutination of allergen gold NPs in the detection of the proper immune response provided good agreement with ELISA data. An immunomagnetic dab ELISA approach using *T. gondii* IgG polyclonal antibodies bundled with attracting NPs to capture circling surface antigen 1 yielded superior results than sandwich ELISA. Using NPs to target diseased macrophages as a stand-alone treatment for toxoplasmosis is a useful and well-known method. In experimental animals, zinc nanoparticles were examined separately and in combination for in vivo toxoplasmosis treatment [17–19]. The interaction of nanoparticles with immune system components is the subject of research interest. Nanoparticles can be tailored to escape immune system detection or to improve or inhibit immune responses selectively. When nanoparticles reach the body, they will very certainly interact with cells. When a nanoparticle interacts with the immune response, it may be used to create vaccinations, pharmaceutical delivery, antigens, or therapies for inflammatory and autoimmune illnesses, among other things. Toxoplasmosis patients' sera will be tested for the presence of research lab zinc (ZnO) nanoparticles, which will be used to assess the impact of certain immune proteins [20–24].

## 2. Materials and Method

### 2.1. Preparation of Zinc Oxide Nanoparticles

Surabhi Siva Kumar et al [25] described a simple precipitation approach for synthesizing ZnO nanoparticles, which was used in this investigation. To make ZnO nanostructures, zinc sulfate heptahydrate and sodium hydroxide were utilized as precursors [26]. The powder generated using the foregoing process was calcined for 2 hours at various temperatures, including 400°C, 600°C, and 800°C.

### 2.2. Sample Collection

In this case-control research, 25 women aged 17 to 26 years, including eight pregnant women, with no clinical problems, took part. From January 2017 to November 2018, blood samples were collected with the authorization of authorities in the Government fever hospital in Guntur, India, and informed consent was obtained from each patient for the purposes of the current investigation. This study included healthy women around the age of 21 as the control group. Participants filled out demographic surveys and were given information papers. After that, 2.5 mL of whole blood was taken, and sera were analyzed for proteins according to usual machine learning. 2.5 mL of venous blood was taken from each sample, deposited in a plane tube, and left to clot for 20 minutes at room temperature before being centrifuged for 15 minutes at 2000 rpm. The serum that resulted was maintained at −20°C until it was used. The activity of serum protease was assessed using casein as a substrate, and the specific activity of protease was represented as mol/g of protein, according to the test machine learning. The Biuret colorimetric machine learning was used to determine the total protein in the serum. IgA, IgG, and IgM were measured using ELISA.

### 2.3. UV-Visible Studies

A spectrophotometer (Unicam UV5-220) was used to perform UV-vis spectral analysis on the produced Zn NPs in the range of 300–800 nm one hour after manufacture, with a quartz cuvette containing water as the reference.

### 2.4. SEM Analysis

Scanning electron microscopy was used to examine the produced samples (SEM). The optical characteristics of ZnO nanostructures were studied, and an attempt was made to connect the optical characteristics of ZnO with shape and crystallite size.

### 2.5. Characterization by SEM-EDX

SEM was used to examine the compounds' structure and morphology. A Philips XL 30 ESEM scanning electron microscope (FEI-Philips Company, Hillsboro) with an EDX analyzer was used to capture SEM pictures of the materials.

### 2.6. Statistical Analysis

The data collected were analyzed with the SPSS software version 11. The data were expressed as mean ± SD.

### 2.7. Ethics Statement

Written consent was obtained from each patient, and ethics approval was obtained from the Ethical Committee of the Machine Centre.

### 2.8. Immunological Study

Using an ELISA kit, interferon gamma (INF) was detected in the serum of patients treated with both ZnO NPs kept at −20°C (Interferon Gamma Elisa kit, Sigma-Aldrich, RAB0520). The assay was carried out according to the manufacturer's instructions. The spiral immunological diffusion approach of Mancini was used to complete the quantitative measurement of immunoglobulins (IgG, IgA, and IgM). ZnO nanoparticles colloidal solution was employed as nanoparticles in this investigation. To get closer to in vivo settings and make it easier to observe an effect, the way of life should be followed for at least 3 days to allow for a few cycles of multiplication.

## 3. Results and Discussion

We use chemical approaches to produce nanoparticles with improved particle characteristics as part of our research program, which helps manage the surface energy. The following procedures were used to characterize the functionalized particles.

### 3.1. UV-Vis Analysis of ZnNPs

The UV-vis absorption spectra of produced ZnNPs at various calcination temperatures are shown in Figure 1 (400, 600, and 800°C). At calcinated temperatures of 400, 600, and 800°C, the absorption peak of ZnNPs was recorded at 366, 366.8, and 367.0 nm, respectively. Because quantum confinement decreases with increasing particle size, the peak absorption wavelength shifts red as temperature rises. The electronic transition from the deep level of the valence band to the conduction band causes these peaks. The variance in UV-vis absorption peaks among ZnNPs is owing to differences in size and shape caused by a range of precursors.

### 3.2. SEM-EDX Analysis

Figure 2(a) shows the SEM pictures of the samples. The morphologies of ZnO vary as the temperature of calcination rises. When calcined at 400°C and 600°C, the samples become nanoflakes, which are then transformed into particles when calcined at 800°C. The agglomerations of particles are substantially less in this way of production, as shown by SEM pictures of ZnO samples.  Figure 2(b) shows spherical-shaped nanoparticles in high-resolution SEM images (3600x, 3800x, and 3700x) of ZnO calcined at 400°C, 600°C, and 800°C. The energy-dispersive spectra of SEM-EDS examination of the samples (Figure 2(a)) clearly shows that the sample made using the above procedure comprises pure ZnO phases. According to the SEM research, the average crystallite size was 42 nm, 37 nm, and 32 nm at 400, 600, and 800°C, respectively.

### 3.3. Nanoparticles Therapy to Humans Affected with Toxoplasmosis

25 patients visited the GFH clinic's toxoplasmosis outpatient service during the pathogenic research period. Based on serology, 16 of them had acute infection with *Toxoplasma gondii*. At the service, the majority of patients were nonpregnant women (64 percent, 16/25) and four were pregnant women (50 percent, 4/8). All of the patients were 20.9 years old on average (median 22.5; SD 11.67).  Figure 2(b) shows the results. It was significantly higher in the pregnant group (*t* = −6.34; *p*0.05). Many pregnant women who were sent to our clinic tested positive for antitoxoplasmosis IgM but negative for IgG, indicating that they had previously been infected but not necessarily recently. Given that toxoplasmosis serology is a regular process in prenatal care in India, this fact indicates that certain pregnancy-related providers are unable to appropriately interpret a serological test, resulting in a false or questionable diagnosis [27]. The average serum monoclonal antibodies in patients and healthy controls are presented in Table 1.

### 3.4. Immunological Results

Table 2 shows the mean INF-*γ* concentrations in each of the subgroup. In general, all infected patients who received NPs had higher INF-*γ* levels. This was particularly noticeable in individuals who were given ZnNPs. Table 2 indicates the concentrations.

## 4. Discussion

Study problem: it has been discovered via epidemiological research that *T. gondii* infection is widespread. Considering that *T. gondii* may infect up to one-third of the world's population, discovering a safe and effective therapy is a big accomplishment.

Traditional therapy is still hampered by major side effects, despite the fact that a variety of approaches have been developed in an attempt to establish an efficient and well-tolerated therapeutic regimen. In the hunt for innovative machine learningto overcome the disadvantages of past treatment regimens, NPs are being employed as experimental therapeutics against toxoplasmosis. To our knowledge, this is the first trial to evaluate ZnNPs as a preventative and therapeutic medication against experimental toxoplasmosis. Previous research has employed NPs as delivery vehicles for medications or vaccinations to boost therapeutic effectiveness. NPs have been employed as a treatment machine learning in various studies. In the lab, turmeric, CS, and AgNPs were all utilized to treat giardiasis. AgNPs and coupled ZnNPs produced the greatest outcomes. Furthermore, gold nanosphere/antibody conjugates were found to be efficient in treating toxoplasmosis in mice. IFN-*γ* is a crucial cytokine that aids the host's defense against intracellular infections. Toll-like receptors (TLRs) recognize pathogens and cause natural killer and T-cells to produce interferon-*γ* (IFN-*γ*). As a result, because IFN-*γ* is an important immunological mediator, it has to be examined. In the current study, the level of IFN-*γ* was increased after infection with *Toxoplasma*. As a result of ZnNPs' increased immunity, the highest level of IFN-*γ* was achieved after their administration. This was more noticeable in ZnNP-treated people (Table 2). Our findings resembled those of Chen et al. [28], who discovered that toxoplasmosis elicited a significant cellular immunological response, with strong IFN-*γ* and IL-2 production associated with a Th1 response. According to Yan et al. [29], AgNPs are also a powerful immune system booster (2012). They act as a powerful adjuvant, stimulating both Th1 and Th2 immune responses. People also attract leukocytes, raise inflammation markers in the abdominal cavity (TNF-a and IFN-*γ*), and upregulate MHC II molecule production in peritoneal macrophages. As a result, ZnNPs showed promising IFN-*γ* concentration findings, with statistically significant agreement between all tests (Table 1). The consequences of parasite load decrease in tissues are clarified by the increase in IFN-*γ* expression in response to AgNPs.

## 5. Conclusion

Although toxoplasmosis is normally a benign and identity condition, late and permanent lesions, such as *T. gondii*, can arise. As a result, acute instances may need to be treated and monitored in order to reduce the hazards associated with such lesions. Even after initial illness and remission, machine personnel must be aware of this parasite and its repercussions. As a result of the findings given in this work, ZnNPs appear to be potential medications for parasite eradication. The modest dose took advantage of their strong protection, lowering the negative side effects and toxicity.

## Figures and Tables

**Figure 1:** UV-vis absorption spectra of ZnNPs at different temperatures.

**Figure 2:** (a): SEM image of ZnNPs calcined at temperature 400°C, 600°C, and 800°C. (b): EDX spectra of ZnNPs calcined at 600°C.

**Table 1:** Serum immunoglobulins (Ig), hemoglobin level, and serum proteins in patients and controls in acute toxoplasmosis before interaction with ZnO nanoparticles.

Parameter tested	Tested group	Tested nos.	Mean ± SD	*p* value
IgA	Patients	25	220.67 ± 12.16	0.194
	Control	20	97.6 ± 22.34	0.237

IgM	Patients	25	267.08 ± 10.36	0.289
	Control	20	167.31 ± 7.61	0.323

IgG	Patients	25	1364.07 ± 6.92	0.395
	Control	20	1401.07 ± 2.37	0.481

Hemoglobin (g/dl)	Patients	25	9.14 ± 1.24	0.477
	Control	20	9.64 ± 1.62	0.481

Total protein (g/dl)	Patients	25	6.07 ± 2.67	0.486
	Control	20	5.97 ± 1.66	0.491

Albumin (g/dl)	Patients	25	4.67 ± 2.02	0.496
	Control	20	4.06 ± 1.68	0.417

Globulin (g/dl)	Patients	25	2.07 ± 1.80	0.350
	Control	20	2.02 ± 1.67	0.294

Protease activity (*µ*mol/L)	Patients	25	684.27 ± 61.37	0.247
	Control	20	651.33 ± 50.63	0.207

**Table 2:** Mean concentration of INF-*γ* in pg/ml in healthy persons and patients treated with ZnNPs after 4 days.

Group name	Healthy persons	ZnNPs immunized group
Concentration	98.5	398

## Data Availability

The data used to support the findings of this study are included within the article.
